The article "Mental Health Evaluation Based on Visual Analysis Technology" was retracted in 2023. Reasons: suspected computer-generated content; unreliable results or conclusions; concerns about the data; concerns about the results or conclusions.

# Mental Health Evaluation Based on Visual Analysis Technology

**DOI:** 10.1155/2022/6706698

**Published:** 2022-03-08

**Authors:** Weifeng Kong

**Affiliations:** Department of Basic Courses, Jiyuan Vocational and Technical College, Jiyuan 459000, China

## Abstract

In order to solve the problems existing in the current mental health assessment system and how to better help individuals analyze their mental health, propose a mental health assessment method based on visual analysis technology; through the study of mental health assessment methods, use the SCL-90 symptom self-rating scale as the mental health assessment scale of this article. Combined with the conceptual design proposed in this article, realize a mental health assessment based on visual analysis technology. The system conducts visual analysis of personal current data and historical data and helps users understand their current mental health. Evaluate the system through user surveys and system quality, and the feasibility and practicability of this method are verified.

## 1. Introduction

With the increasingly fierce social competition, the incidence of psychological disorders among college students is on the rise. Research shows that at present, the incidence of psychological problems among college students is between 10% and 30%; mental health is not optimistic, psychological problems; it has become one of the main reasons for college students to drop out and commit suicide in our country. At present, all domestic colleges and universities have established psychological counseling departments, conduct mental health education, and provide consulting services for college students [1]. According to the investigation, in order to understand the psychological condition of freshmen in colleges and universities, the mental state scale is generally used: carry out census and statistics through questionnaire surveys, screen out students with warning conditions, counselors at all levels and specialized psychological educators will further screen and judge, and intervention treatment for students with serious psychological problems [2]. This method aims to prevent psychological crisis events, and health promotion and preventive intervention are more passive. Psychological research believes that personality and mental state are closely related, and the former has a significant predictive effect on the latter [3].

Today, with the rapid development of the Internet, information technologies such as big data and cloud computing have been integrated into all aspects of people's lives; people generate a lot of data every day, and data from a simple processing object become a basic resource. People want to get the knowledge and wisdom contained in the data; you need to dig out the hidden information behind the data; as a result, visual analysis emerged as a new analytical method. Visual analysis provides fast, testable, and understandable assessments, and it can explore unknown content and detect expected information. Visual analysis is a new analysis method; it is used in the field of mental health; under the influence of visual analysis, many characteristics of mental health are beginning to show up, but research on this aspect is still in its infancy. Simultaneously showing the mental state and personality characteristics through visual analysis, there are relatively few research studies on mining potential information; visualization converts data into visual elements such as graphics, symbols, colors, and textures that are easily perceivable by the human eye, and it can effectively enhance the efficiency of feature recognition and efficiently transmit valuable information [4–6].

Based on this research, the author introduces the current research status of visual analysis technology in psychology, analyze the key points and difficulties in the current application of visual analysis technology in the direction of mental health, and points out the existing problems of the current mental health evaluation system research.

## 2. Research Methods

### 2.1. Visual Analysis Technology and Mental Health Assessment

#### 2.1.1. Visual Analysis Technology Research

In this era of big data, people's daily lives are generating a lot of data, so how to use these data reasonably, solve the diversity and complexity of data, exploring the hidden value in data have become a very hot research direction [7, 8]. The starting point of the standard process of visual analytics is the input data, the end point is to extract knowledge, and the application should include the four characteristics of intuitiveness, relevance, artistry and interactivity.  Figure 1 shows the standard process of visual analytics.

#### 2.1.2. Scientific Visualization

Scientific visualization was originally called visualization in scientific computing and refers to visualization as an integral part of scientific computing. Research focuses on scientific visualization and how to display scientific data with geometric attributes in a three-dimensional data field truly and quickly; the image quality is the core issue considered. Scientific visualization is mostly used in the simulation of the three-dimensional real world; it can be divided into three parts: scalar field visualization, vector field visualization, and tensor field visualization.  Figure 2 shows the basic design process of scientific visualization.

### 2.2. Mental Health Assessment Methods

#### 2.2.1. SCL-90 Symptom Self-Rating Scale

The SCL-90 symptom self-rating scale is currently one of the most famous mental health test scales; it is widely used in various mental illness clinics. The SCL-90 symptom self-rating scale contains a total of 90 self-evaluation items, and according to the content detected by each assessment item, 90 self-assessment items are divided into 10 factors. Among them, 10 factors reflect the mental health of the testee in 10 aspects; the 10 factors and their reflections are given in Table 1.

Evaluation time of the SCL-90 symptom self-rating scale as the “current” or the actual feeling of the subject in the “last week;” for the specific evaluation of each item, participants will define the “light, medium, and heavy” in the scoring system according to their own experience. Each item adopts a 5-level scoring system, as given in Table 2.

The results of the SCL-90 symptom self-rating scale are divided into the total score of the participant and analysis of factors and individual items with “symptoms;” the specific explanation about each result item is given in Table 3. Among them, each of the 10 factors is equally divided; they can reflect the subject's mental health in 10 aspects; participants can also understand the distribution of their total scores through factor averaging.

In actual testing, usually in the results of the SCL-90 symptom self-rating scale, compare and analyze with the norms that scholars have researched; the author uses the standard norm used by the school's psychological counseling studio to evaluate the test results.  Table 4 provides the evaluation and analysis of the results of the SCL-90 symptom self-rating scale, the standard norm used.

### 2.3. Feature Selection Algorithm

#### 2.3.1. Filtering Method

The following introduces several common algorithms in the filtering method; among them, the variance selection method is based on each feature, and the divergence of the target to select features, such as the correlation coefficient method, the chi-square test, and the maximum information coefficient rule; the feature is selected according to the correlation between each feature and the target [9, 10].

*(1) Variance Selection Method*. The variance is used to reflect the degree of deviation of the random variable from the expected value. When using the variance selection method, first, calculate the variance of each feature according to the variance formula. Second, set different threshold selection rules according to different needs analysis. Finally, according to the set threshold selection rules, the features that meet the rules are selected. The calculation of variance is

(1) $$\begin{array}{c} s^{2}=\frac{1}{n-1}{\sum_{i=1}^{n}\left(x_{i}-\bar{x}\right)}^{2}, \end{array}$$

where *s* represents the standard deviation, *n* represents the sample size, *x*_*i*_ represents an individual, and $\bar{x}$ represents the average number of samples.

*(2) Correlation Coefficient Method*. The correlation coefficient is generally represented by the letter *r*; when using the correlation coefficient method, first of all, calculate the correlation coefficient of each feature to the target value according to the correlation coefficient formula. Second, calculate the *P* value of the correlation coefficient of each feature; finally, the feature is selected based on the *P* value calculated from each feature and the target value. The calculation of the correlation coefficient is

(2) $$\begin{array}{c} r\left(X,Y\right)=\frac{\text{Cov}\left(X,Y\right)}{\sqrt{\text{Var}\left[X\right]\text{Var}\left[Y\right]}}, \end{array}$$

where Cov(*X*, *Y*) represents the covariance of *X* and *Y*, Var[*X*] represents the variance of *X*, and Var[*Y*] represents the variance of *Y*.

*(3) Chi-Square Test*. The chi-square test is used to detect the degree of deviation between the actual observation value and the theoretical inferred value. The chi-square value has a linear relationship with the degree of deviation between the actual observation value and the theoretical inferred value; the smaller the chi-square value, the smaller the degree of deviation and vice versa; the greater the chi-square value, the greater the degree of deviation; when the chi-square value is small, it tends to conform. When the actual observed value is in full agreement with the theoretically inferred value, the chi-square value is 0. The calculation of test statistics is

(3) $$\begin{array}{c} x^{2}=\sum \frac{{\left(f_{o}-f_{e}\right)}^{2}}{f_{e}}, \end{array}$$

where *f*_*o*_ represents the observed frequency and *f*_*e*_ represents the expected frequency.

*(4). Mutual Information and Maximum Information Coefficient Method*. The mutual information method is used to measure the mutuality between two variables, and its calculation is

(4) $$\begin{array}{c} I\left(X;Y\right)=\sum_{x\in X}\sum_{y\in Y}p\left(x,y\right)\log\frac{p\left(x,y\right)}{p\left(x\right)p\left(y\right)}, \end{array}$$

where *p*(*x*, *y*) represents the joint distribution of two random variables (*X*, *Y*) of observation frequency, *p*(*x*) represents the marginal distribution, and *p*(*y*) force represents the marginal distribution.

#### 2.3.2. Embedding Method

Embedded refers to the use of algorithms and models to train features; the feature is selected according to the weight coefficient of each feature. The embedding method mainly includes the feature selection method based on the regular term and the feature selection method based on the tree model. Here, mainly select the feature selection method based on regular term.

Regularization refers to adding additional constraints or penalties to the existing model (loss function), in order to prevent overfitting and improve generalization ability [11]. For linear regression models, the model using *L*1 regularization is called Lasso regression, the model using *L*2 regularization is called ridge regression. The main purpose of *L*1 regularization is to generate sparse models, that is, the sparse weight matrix; it adds the *L*1 norm of the coefficient vector *w* as a penalty term to the loss function; since the regular term is nonzero, this forces the coefficients corresponding to those weak features to become zero. The loss function of *L*1 regularization is

(5) $$\begin{array}{c} J=J_{0}+\alpha \sum_{w}\left|w\right|, \end{array}$$

where *J* represents a function with an absolute value symbol, *J*_0_ represents the original loss function, and *α* represents the regularization coefficient.

Make $L=\alpha \sum_{w}\left|w\right|$; then, *J*=*J*_0_+*L*, where *L* is a constraint on *J*_0_; the task of machine learning is to find the minimum value of the loss function (*J*) through some methods. The loss function of Lasso regression is

(6) $$\begin{array}{c} \underset{w}{\min}\frac{1}{2n_{\text{samples}}}{\left\|X_{w-y}\right\|}_{2}^{2}+\alpha {\left\|w\right\|}_{1}, \end{array}$$

where *w* represents the coefficient of the feature.

The main purpose of *L*2 regularization is to prevent the model from overfitting; it adds the *L*2 norm of the coefficient vector *w* as a penalty term to the loss function. The loss function of *L*2 regularization is

(7) $$\begin{array}{c} J=J_{0}+\alpha \sum_{w}w^{2}. \end{array}$$

Compared with *L*1 regularization, *L*2 regularization tends to make the weight of the feature as small as possible. Take the gradient descent method in linear regression as an example to illustrate how *L*2 regularization obtains parameters with small values. Suppose the parameter to be solved is *θ* and *h*_*θ*_(*x*) is a hypothetical function, then the cost function of linear regression is

(8) $$\begin{array}{c} J\left(\theta \right)=\frac{1}{2m}\sum_{i=1}^{m}\left(h_{\theta }\left(x^{\left(i\right)}\right)-y^{\left(i\right)}\right). \end{array}$$

### 2.4. Research on Mental Health Assessment Methods Based on Visual Analysis Technology

#### 2.4.1. Data Processing

The purpose of data processing (DataProcessing) is to extract from a large amount of messy data, filter, and derive valuable and meaningful data [12]. The author collects, stores, retrieves, processes, transforms, and transmits SCL-90 symptom self-rating scale data as basic data.

#### 2.4.2. Color Scheme and Interactive Functions

An excellent visualization system is inseparable from a reasonable color scheme and good user interaction; the color scheme affects people's understanding of the visualized view through color; interaction can help users better participate in the understanding and analysis of data. The author system applies the HSL color space to each visualization view, such as scatter graphs, line graphs, word clouds, and stack graphs.  Figure 3 shows the comparison effect before and after color matching of the stack map for analyzing the national data.

## 3. Result Analysis

In order to make visual analysis technology better used in mental health assessment, the author has conducted many explorations. When designing the visualization program, based on the SCL-90 symptom self-rating scale, through the study of the existing mental health assessment system, a variety of visualization schemes are explored and analyzed, and each visualization scheme is described in detail [13].

### 3.1. The First Exploration of Visualization Schemes

The visualization scheme designed for the first time is shown in Figure 4. The existing mental health assessment systems all evaluate users in the form of text scales; then, when the user submits the scale, the system calculates and analyzes the scale data and give the results shown in the “Evaluation Results” block in Figure 4. Such results are not easy to understand directly, and it is not clear what state the user's total evaluation score is in and what the results of each factor are. The author compares the calculated user results with the standard norm and tell the user the extent of the result directly in a visual way.

### 3.2. Exploration of the Second Visualization Scheme

Analyze and improve the problems in the first visualization scheme; the result after the first improvement is obtained, as shown in Figure 5. The improved visualization scheme divides the interface into 6 parts, through the interaction analysis between different visualization views, in order to enhance users' understanding and analysis of the evaluation data. Besides improved visualization scheme, users are required to complete a complete SCL-90 symptom self-assessment questionnaire before they can view their own assessment results, and it relatively reduces the impact of the visual view on the user when the user fills in the questionnaire.

The matrix tree diagram is an extension of the hierarchical layout; according to the data, the area is divided into a collection of rectangles [14, 15]. The tree diagram starts from the root node, and how many rectangles are divided into corresponding subnode data and the area of the rectangle usually correspond to the attributes of the node. Each rectangle continues to be divided according to the child nodes of the corresponding node, until only leaf nodes are left. As shown in Figure 6, the tree on the left can be represented by the tree diagram on the right.

Figures 7 and 8 show the use of matrix tree diagrams to replace the original packed diagram and Sankey diagram, combine line chart and column chart, and analyze the SCL-90 symptom self-rating scale data entered by the user once, the colors of the questions and factors in the matrix tree diagram, line graph, and histogram correspond to the colors on the right side of the matrix tree diagram. Among them, the matrix tree diagram divides and categorizes each problem; each factor contains several questions represented by the small matrix contained, whether the problem is in a normal state, use color to distinguish, normal problems are represented in gray, and problems in a subhealth state are represented in the same color as the respective factors.

### 3.3. The Mental Health Assessment System Architecture Based on Visual Analysis Technology

Software architecture refers to the abstract design of software; it is a systematic sketch; two commonly used software development architectures are C/S (client/server) architecture and B/S (browser/server) architecture [16, 17]. The C/S architecture is a two-tier architecture, which is divided into two tiers: client and server; the first layer is the user presentation layer that receives and processes user requests on the client side and the second layer is the database layer for database operations, also known as the service layer. The user sends a request to the server through the client; the server receives the request and processes it and then returns the processed result to the client.  Figure 9 shows the schematic diagram of a two-tier C/S architecture.

The B/S architecture is an improvement to the C/S architecture; it is a three-tier architecture divided into client (presentation layer), application server (business logic layer), and database server (data storage layer).  Figure 10 shows a schematic diagram of a three-layer B/S architecture.

According to the demand analysis of the system, the mental health assessment system based on visual analysis technology is developed using B/S architecture; based on Web implementation, users can understand and analyze personal mental health assessment data through a browser and can interact with the data through the interface [18, 19].

### 3.4. User Evaluation

The author made statistics on the survey results from four aspects: beauty, accuracy, practicality, and user experience.  Figure 11 shows the statistical results of user feedback. Through the survey results can be found that the mental health assessment system of visual analysis has reached 23 and 27 in practicability and accuracy, and the response is good, regarding the aesthetics, and usage of the system as low as 15 is relatively general, and there are still many areas that need to be improved.

## 4. Conclusion

The author takes the development of the personality of college students as a starting point, researching and summarizing the research on the mental health and personality of college students in related fields of psychology and choose to use the mental health self-rating scale SCL-90 for data collection and analysis. Effectively evaluate the differences in the analysis results of multisource questionnaires through geometric spatial difference metrics and use color mapping to effectively guide users to pay attention to individual students whose analysis results are uncertain, so as to realize the comprehensive judgment and tracking analysis of mental health status. Effectively integrate the user's prior knowledge, judging the mental health of college students through the use of feedback by relevant researchers; this method is visually displaying data, mining hidden information, and guiding decision-making, and other aspects have both the theoretical value and practical value.

## Figures and Tables

**Figure 1:** Visual analytics standard process.

**Figure 2:** The basic design process of scientific visualization.

**Figure 3:** Comparison of effects (a) before and (b) after stacking color matching.

**Figure 4:** The first visualization scheme diagram.

**Figure 5:** The first revision of the visualization scheme.

**Figure 6:** Tree data structure and tree diagram representation.

**Figure 7:** The factor line graph of the second visualization scheme.

**Figure 8:** The second time visualization scheme problem histogram.

**Figure 9:** Schematic diagram of two-tier C/S architecture.

**Figure 10:** Schematic diagram of three-layer B/S architecture.

**Figure 11:** User feedback statistics.

**Table 1:** Explanation of each factor of the SCL-90 symptom self-rating scale.

Factor item	Reflect symptoms
Somatization	Mainly reflects the subject's physical discomfort
Obsessive-compulsive symptoms	Mainly reflect the compulsive psychology of subjects in life and may show some behavioral signs of cognitive impairment
Interpersonal sensitivity	It mainly reflects the subjects' inferiority complex, negative expectations, and bad self-suggestion and uncomfortable feelings in interpersonal communication.
Depression	It mainly reflects the depressed emotions and mood of the subjects, decreased interest in life, and loss of vitality. In addition, it also includes the thought of death and the idea of suicide.
Anxiety	Mainly reflect the subject's irritability, restlessness, nervousness, and the physical symptoms produced by this emotion
Hostility	It mainly reflects the hostile emotions of the subjects in the three aspects of thoughts, feelings, and behaviors; this includes tests for boredom, falling objects, and uncontrollable temper.
Fear	It mainly reflects the horror psychology of the subjects on traveling, public places, open spaces, crowds, and vehicles.
Paranoid	Mainly reflect the subjects' delusions, suspicions, passive experiences, and exaggerated projective thoughts
Psychotic	It mainly reflects whether the subject has a variety of acute symptoms and behaviors, mainly including the detection of schizophrenic items such as auditory hallucinations, thought transmission, and feelings of insight.
Other	Mainly reflect the subject's sleep and diet

**Table 2:** Explanation of the degree of each item of the SCL-90 symptom self-rating scale.

Project level	Degree explanation
No	Participants feel that they have no such problem
Very light	Participants feel that they have this symptom, but there is no actual effect or the effect is slight
Moderate	Participants feel that they have this symptom and have a certain degree of influence
Partiality	Participants feel that they have this symptom, and have a considerable impact
Serious	Participants feel that the frequency and intensity of the symptoms are very severe

**Table 3:** Explanation of each evaluation result item of the SCL-90 symptom self-rating scale.

Result item	Interpretation of results
Total symptom index	Reflect the overall mental health of the subjects
Number of daily items	Reflect how many items the subject feels “symptomatic”
Number of negative items	Reflect how many items the subject feels “asymptomatic”
Positive symptoms are evenly divided	What is the extent of the “symptomatic” items felt by the subjects
All factors are equally divided	Reflect the subjects' mental health in 10 aspects

**Table 4:** Reference norm of the SCL-90 symptom self-rating scale.

Factor item	Norm	Factor item	Norm
Somatization	1.26 ± 0.37	Fear	1.12 ± 0.31
Obsessive-compulsive symptoms	1.51 ± 0.47	Paranoid	1.32 ± 0.46
Interpersonal sensitivity	1.54 ± 0.41	Psychotic	1.18 ± 0.31
Depression	1.40 ± 0.48	Total score	118.85 ± 37.65
Anxiety	1.28 ± 0.32	Total average score	1.33 ± 0.32
Hostility	1.37 ± 0.45	Symptoms are evenly divided	2.50 ± 0.48

## Data Availability

The datasets used and/or analyzed during the current study are available from the corresponding author upon request.
